# Impact of YouTube Advertising on Sales with Regression Analysis and Statistical Modeling: Usefulness of Online Media in Business

**DOI:** 10.1155/2021/9863155

**Published:** 2021-09-07

**Authors:** Yang Zhou, Zubair Ahmad, Hassan Alsuhabi, M. Yusuf, Ibrahim Alkhairy, A. M. Sharawy

**Affiliations:** ^1^School of Journalism and Communication, Xiamen University, Xiamen, Fujian Province, China; ^2^Department of Statistics, Yazd University, P.O. Box 89175-741, Yazd, Iran; ^3^Department of Mathematics, Al-Qunfudah University College, Umm Al-Qura University, Mecca, Saudi Arabia; ^4^Department of Mathematics, Faculty of Science, Helwan University, Helwan, Egypt; ^5^Department of Mathematical and Natural Sciences, Faculty of Engineering, Egyptian Russian University, Badr, Egypt

## Abstract

Computer technology plays a prominent role in almost every aspect of daily life including education, health care, online shopping, advertising, and even in homes. Computers help to make daily tasks much easier and convenient. Among social media, YouTube is a well-known social sharing networking service. As more and more people join social media and become everyday users, brands have also increased their online engagement. However, it is still unclear how to effectively measure value and return on advertising using social media. As of 2021, more than 31 million YouTube channels around the globe have been opened. In this paper, we consider YouTube advertising to check its effectiveness and benefits gained. Certain statistical tools are adopted to measure the extent of advertising benefits and their correlation in creating effective advertising campaigns on YouTube. Simple linear regression analysis is performed on the data representing the YouTube advertising budget of a company and the sales data of that company. Furthermore, we develop a new statistical distribution to provide the best description of the YouTube advertising data. The result of this research shows that YouTube is an effective medium for advertising and has a strong relationship with sales.

## 1. Introduction

Marketing is a collection of all those strategies that a company adapt to convey their messages or brands to their concerned audience. It has a key role in motivating the consumers to buy the company's brand or product [1]. Marketers can promote their brands directly to businesses (also called B2B marketing) or direct their products to consumers (also called B2C marketing). Basically, marketing has four principles (4Ps) such as (i) Product (P1), (ii) Price (P2), (iii) Place (P3), and (iv) Promotion (P4). These 4Ps are collectively known as marketing matrix [2].

The P1 refers to the company's services or products offered to their consumers. It deals with the warranty, packaging, appearance, quality, and so on. The P2 refers to the setup of the product's price. It not only deals with the selling price but also deals with the payment arrangement, discount, and credit terms. The P3 deals with the identification of the location where the company's product/service is made or distributed. The P4 includes the activities to influence the customer's decision and make the business known to them [3].

In the literature, numerous strategies (online and print mediums) have been suggested for marketing. However, among the available strategies, online advertising or online marketing is the most effective to reach the maximum audience. A number of venues are available for online marketing such as Facebook, YouTube, Twitter, Flickr, Pinterest, and Instagram [4]. Among the possible venues for online marketing, YouTube is one of the most effective platforms for online marketing (see Djafarova and Matson [5]; Pleyers and Vermeulen [6]; Semeradova and Weinlich [7]; Acikgoz and Burnaz [8]; and Al-Maroof et al. [9]).

YouTube is the second most popular SE (search engine) around the globe and provides an effective way of advertisement to capture consumer's attention. Around the mid of 2005, YouTube shared its first video, and since that grew rapidly. By March 2019, YouTube crossed a number of 1.5 billion active monthly users. Due to many active users, it attracted the attention of different business firms to spend more and more on advertising through YouTube. According to Abdelkader [10], the top hundred (100) advertisers of YouTube have increased their spending budget by over 60% annually.

In this paper, we use the YouTube medium as an advertising tool and test its impact on the sales of a company. To check its usefulness, a widely used statistical technique called SLRM (simple linear regression model) is adopted. In this regard, we test a claim (also called a hypothesis) using two different statistical tests, such as *t*-test and *F*-test. To carry out the statistical analysis, the NH (null hypothesis) *H*_0_ and AH (alternative hypothesis) *H*_1_ are formulated as *H*_0_ = *YouTube advertising has no significant relationship with sales* vs.*H*_1_ = *YouTube advertising has a significant relationship with sales*.

Besides the regression analysis, a new SD (statistical distribution) is proposed to model the YouTube advertising data. The new SD is called a HTBPT-Lomax (heavy-tailed beta power transformed Lomax) distribution. The HTBPT-Lomax is very flexible and possesses the HT (heavy-tailed) characteristics.

## 2. Methodology

In the practice of economic studies, regression analysis (RA) is a prominent technique that helps econometricians to know about how the dependent variable changes in relation to changes in independent variables [11]. In simple words, the RA helps to understand how the likelihood of the sale (dependent variable) is impacted by price or quantity purchased (independent variables) (see Nunez et al. [12]). There are main two types of RA, called (i) simple linear RA (SLRA) and (ii) multiple linear RA (MLRA).

In this work, we focus our study on SLRA, only. The SLRA assists to measure the relationship between *Y* (the output of the regression model) and an explanatory variable *X* (the input of the regression model). The simple linear regression model (SLRM) is defined by

(1) $$\begin{array}{c} Y=\beta_{0}+\beta_{1}X+\varepsilon , \end{array}$$

where

- *Y* represents the outcome of the model that is what we are trying to predict.
- *X* represents the input of the model that helps in predicting *Y.*
- *β*_0_ is called the intercept of the model. If *X*=0 (it means that *X* has no effect on *Y*), then *Y*=*β*_0_.
- *β*_1_ is called the slope of the model and represents per unit changes in the outcome of the regression model.
- *ε* represents the residual error term (RET) having a mean or an average value of 0.

## 3. Regression Analysis

The RA is widely used for two different conceptual purposes. First, regression analysis is used for prediction and forecasting, where its uses are closely related to the field of machine learning. Second, regression analysis is used to establish a causal relationship (CR) between *X* (predictor variables) and *Y* (response variable).

The RA has many applications in insurance, finance, and business, among others. In business and finance, RA is used to calculate the Beta (return volatility relative to the entire market) for a stock. The RA can also be used to predict the returns of business or predict business performance. This section offers RA to predict the *Y* (sale) based on the predictor variable (YouTube advertising).

### 3.1. Simple Linear Regression Model

The SLRM to explain the relationship between YouTube advertising and sales is given by

(2) $$\begin{array}{c} Y=\beta_{0}+\beta_{1}\text{YouTube}+\varepsilon . \end{array}$$

After performing the regression technique, we observe that the value of *β*_0_ is 4.84708, which represents the predicted/estimated dollar sales (in thousands) for spending no advertising budget on the YouTube medium. Henceforth, for spending nothing on the YouTube advertising, the expected sale (ES) is 4.84708*∗*1000=$4847. The slope of the model provided in equation (2) is 0.04802 indicating 48 (1000*∗*0.04802) units increment in the sales. So, spending money on the YouTube medium, the ES is 4.84708+0.04802*∗*1000=52.86708, representing a sale of $52867. Corresponding to equation (2), the fitted regression model is given by

(3) $$\begin{array}{c} Y=4.84708+0.04802\text{YouTube}+\varepsilon . \end{array}$$

A visual display of the relationship between YouTube advertising and sales is provided in Figure 1. The plot obtained in Figure 1 represents a positive relationship. Therefore, spending money on YouTube advertising results an increase in the sale.

### 3.2. Hypothesis Testing

We adopt a well-known statistical procedure (hypothesis testing) to test the significance of YouTube advertising on sales. To carry out the analysis, the null (*H*_0_) hypothesis and alternative (*H*_1_) hypothesis can be formulated as *H*_0_ = YouTube advertising has no significant relationship with sales vs. *H*_1_ = YouTube advertising has a significant relationship with sales.

The standard error (SE) is very useful in performing hypothesis testing to test the regression coefficients (RCs). The SE measures the reliability of the coefficient estimates (CEs) and quantifies how far the CEs vary from the actual average/mean value of *Y*.

### 3.3. *t*-Test

To test *H*_0_, first, we have to find whether the estimate of the regression coefficient *β*_1_ is far from 0 or not. If the SE of the estimate of *β*_1_ is too small, then even a small value of the estimate of *β*_1_ will provide sufficient evidence against *H*_0_. We use the *t*-test to measure how far *β*_1_ is from zero. After implementing the *t*-statistic, the obtained results are provided in Table 1.

The value of the *t*-statistic shows how far the CE is from zero. Relative to SE, a larger value of the *t*-statistic provides evidence against *H*_0_ and indicates that *Y* is associated with *X*. The value Pr(>|*t*|) indicates that the *p* value is greater than the *t*-statistic. The smaller the *p* value, the more chances to reject *H*_0_.

From Table 1, it is obvious that the value of the *t*-statistic (for YouTube advertising) is far from zero, and the *p* value < 0.05 indicate that the value of *β*_1_ is not equal to zero. Based on the above results and discussion, we can obtain that there is sufficient evidence to reject *H*_0_.

### 3.4. *F*-Test

Here, we implement another powerful statistical test (called *F*-test) to check the impact of YouTube advertising on sales. If the value of the *F*-statistic is far from zero, then it is indicating a positive impact of YouTube advertising on sales. As given in Table 2, the value of the *F*-statistic is 99.18. Henceforth, using YouTube advertising medium as a predictor variable to predict *Y* indicates the better model.

The *R* square (*R*^2^) is one of the most powerful/important statistical quantities used for measuring the quality of the model fit, and its values range from 0 to 1. The *R*^2^ deals with the linear relationship between the predictor variable and the response variable. For a particular model, if the value of *R*^2^ is near to 0 (near to 1), it represents the poor fit (the better fit). In this study, the value of *R*^2^ is 0.4366 indicating that the sale can be increased up to 43.66%.

### 3.5. Residuals

In statistics and optimization, the residuals represent the deviation of an observed value of an element and its theoretical value. In regression analysis, the residual is the difference between any data point and the regression line. Sometimes they are also known as an error. An error in this context does not mean that something is wrong with the analysis; it just means that there is an unexplained difference between the observed and theoretical values. In simple words, the residual is the error that is not explained by the regression line.

The residual, represented by *ε*, can also be expressed by an equation. The term *ε* is the difference between observed value *y* and predicted value $\hat{y}$. Mathematically, we have

(4) $$\begin{array}{c} \varepsilon =y-\hat{y}. \end{array}$$

The residual SE measures the quality of the fit of the regression model [13]. In the context of this study, different plots for the behavior of the residual are presented in Figure 2. From Figure 2, we can see that

- The red line in the residual vs. fitted plot (see Figure 2) lies closer to the residual value of 0. Therefore, based on the residual vs. fitted plot in Figure 2, we can say that the residuals of the model are linearly related. Linearity means that the predicted variable in the regression model has a straight-line relationship with *Y.*
- Homoscedasticity is a fundamental assumption of linear regression models. If this assumption is violated, the problem of heteroscedasticity arises. The scale-location plot shows the fact that the residuals satisfy the homoscedasticity property.
- In RA, an observation whose deletion from the data has a significant effect on the estimates of the model parameters is called influential observation. The residual vs. leverage plot shows that there are fewer influential observations.
- The plot of the quantile-quantile (Q-Q) function is a visual approach to check the normality. The Q-Q plot makes an angle of 45° (see Figure 2), which leads to the fact that the residuals are approximately normally distributed.

### 3.6. Outlier Test

In this subsection, we perform the outlier test to detect whether there are outliers in the residual's data or not. After performing the outlier test, we observe that the 23^rd^ observation has the largest error. We can also see that the outlier is present as shown in box plot provided in Figure 3. Furthermore, we check the influential observations by using Cook's distance. Any observation that is far from Cook's distance is known as influential observation. We use the standard cut-off rule of 4/*n* to identify the influential observations. Here, we can see that the 23^rd^ observation is far from Cook's distance, representing the influential observation.

### 3.7. Correlation Test

The correlation test is used to evaluate the association between two or more variables. Here, we have two variables (YouTube advertising and sales); therefore, we use the Pearson correlation analysis approach which measures a linear dependence between two variables. The Pearson correlation coefficient, denoted *r*, is obtained as

(5) $$\begin{array}{c} r=\frac{\sum_{i=1}^{130}\left(\text{Youtube}-M_{\text{Youtube}}\right)\left(\text{Sales}-M_{\text{Sales}}\right)}{\sum_{i=1}^{130}{\left(\text{Youtube}-M_{\text{Youtube}}\right)}^{2}{\left(\text{Sales}-M_{\text{Sales}}\right)}^{2}}, \end{array}$$

where *M*_YouTube_ and *M*_Sales_ are the means of YouTube and sales, respectively. The *p* value (also called significance level) of the correlation can be obtained either by (i) using the correlation coefficient table with degree of freedom: *n-2*, where *n* represents the number of observations of YouTube and sales data or (ii) calculating *t* value, given by

(6) $$\begin{array}{c} t=\frac{r}{\sqrt{1-r^{2}}}\sqrt{n-2}. \end{array}$$

It is worthwhile to note that if the *p* value is <0.05, then the correlation between YouTube advertising and sales is significant. Using the above procedure, we observe that *r*=0.66073, which shows that there is a positive relationship between YouTube advertising and sales (see Figure 4). We also found that the *p* value is 2.2*e* − 16. Since the *p* value is less than 0.05, therefore, we reject the hypothesis of no relationship between YouTube advertising and sales.

## 4. Statistical Modeling

After showing the impact of YouTube advertising in the above sections, we now introduce a new statistical model for analyzing the YouTube advertising data. This section consists of three subsections: (i) the first phase of this section deals with the introduction of the statistical model, (ii) the second subsection deals with the parameter estimation, and (iii) the third section deals with the modeling of YouTube advertising data.

### 4.1. A New Statistical Distribution

The introduction of the new statistical distributions to model real phenomena is a prominent research topic, that is, quite rich and still increasing continuously. Among the applied fields, the statistical distributions play a prominent role to model financial and actuarial data sets. For example, Zhu and Galbraith [14] introduced a generalized asymmetric Student-*t* (GAS-*t*) distribution for analyzing econometric and financial data. Marchant et al. [15] studied the generalized Birnbaum–Saunders (GBS) distribution and analyzed data in management sciences. Nadarajah and Bakar [16] applied new composite models (CMs) to Danish fire insurance data. Theodossiou [17] considered the skewed generalized error (SGE) distribution for financial assets and returns. Bhati and Ravi [18] studied the generalized log-Moyal (GLM) distribution and analyzed the Norwegian fire insurance loss data. Punzo et al. [19] suggested finite mixtures of contaminated gamma (FMCG) for fitting econometric data. Punzo [20] used inverse Gaussian (IGa) distribution for modeling insurance and econometric data. Ahmad et al. [21] proposed a class of claim (CC) distributions and applied it to insurance claim data. Ahmad et al. [22] introduced the Z-Weibull distribution for analyzing the earthquake insurance data. Ahmad et al. [23] introduced new methods for generating heavy-tailed (HT) distributions and analyzed insurance data. Punzo and Bagnato [24] used the Laplace scale mixtures (LSMs) for modeling data related to cryptocurrencies. Tung et al. [25] introduced a new statistical distribution for modeling medical care insurance data. Zhao et al. [26] proposed the Lomax-Claim (LC) model to analyze the financial data. For more details about the usefulness of statistical distributions in applied sciences, we refer to Ahmad et al. [27].

We further carry this branch of distribution theory and introduce a new distribution to model the YouTube advertising data. The proposed model may be called the heavy-tailed beta power transformed Lomax (HTBPT-Lomax) distribution.

The cumulative distribution function (CDF) *U*(*y*; *ξ*) of the Lomax distribution is given by

(7) $$\begin{array}{c} U\left(y;\xi \right)=1-{\left(1+\lambda_{2}y\right)}^{-\lambda_{1}},\;y\geq 0,\lambda_{1},\lambda_{2}>0, \end{array}$$

where *ξ*=(*λ*_1_, *λ*_2_). The respective PDF (probability density function) expressed by *u*(*y*; *ξ*) is

(8) $$\begin{array}{c} u\left(y;\xi \right)=\lambda_{1}\lambda_{2}{\left(1+\lambda_{2}y\right)}^{-\lambda_{1}-1},\;y,\lambda_{1},\lambda_{2}>0. \end{array}$$

Recently, Zhao et al. [28] introduced a new family called heavy-tailed beta power transformed (HTBPT) family of distributions. Its CDF *P*(*y*; *β*, *ξ*) and PDF *p*(*y*; *β*, *ξ*) are given by

(9) $$\begin{array}{c} P\left(y;\beta ,\xi \right)=\beta^{1-U\left(y;\xi \right)}-\beta \left[1-U\left(y;\xi \right)\right],\;y\in \mathbb{R},\beta >0,\\ p\left(y;\beta ,\xi \right)=u\left(y;\xi \right)\left[\beta -\log\left(\beta \right)\beta^{1-U\left(y;\xi \right)}\right],\;y\in \mathbb{R},\beta >0, \end{array}$$

respectively.

Using equation (7) in equation (9), we get the CDF of the HTBPT-Lomax model given by

(10) $$\begin{array}{c} P\left(y;\beta ,\xi \right)=\beta^{{\left(1+\lambda_{2}y\right)}^{-\lambda_{1}}}-\beta {\left(1+\lambda_{2}y\right)}^{-\lambda_{1}},\;y\geq 0,\beta ,\lambda_{1},\lambda_{2}>0. \end{array}$$

The respective PDF is

(11) $$\begin{array}{c} p\left(y;\beta ,\xi \right)=\lambda_{1}\lambda_{2}{\left(1+\lambda_{2}y\right)}^{-\lambda_{1}-1}\left[\beta -\log\left(\beta \right)\beta^{{\left(1+\lambda_{2}y\right)}^{-\lambda_{1}}}\right],\;y>0. \end{array}$$

Different plots of the HTBPT-Lomax PDF *p*(*y*; *β*, *ξ*) are provided in Figure 5. These plots are obtained for *λ*_1_=1.2, *λ*_2_=1, and *β*=1.9 (red line); *λ*_1_=1.2, *λ*_2_=1, and *β*=3.1 (green line); *λ*_1_=1.2, *λ*_2_=1, and *β*=5.5 (black line); and *λ*_1_=1.2, *λ*_2_=1, and *β*=8.2 (blue line).

### 4.2. Estimation

Here, the estimators $\left(\hat{\lambda_{1}},\hat{\lambda_{2}},\hat{\beta }\right)$ of the parameters (*λ*_1_, *λ*_2_, *β*) are obtained. Consider a random sample, say *y*_1_, *y*_2_,…, *y*_*n*_ obtained from *p*(*y*; *β*, *ξ*). Then, corresponding to *p*(*y*; *β*, *ξ*), the log-likelihood function *π*(*λ*_1_, *λ*_2_, *β*) is

(12) $$\begin{array}{c} \pi \left(\lambda_{1},\lambda_{2},\beta \right)=n\;\log\;\lambda_{1}+n\;\log\;\lambda_{2}-\left(\lambda_{1}+1\right)\sum_{k=1}^{n}\log\left(1+\lambda_{2}y_{k}\right)\\ +\sum_{k=1}^{n}\log\left[\beta -\log\left(\beta \right)\beta^{{\left(1+\lambda_{2}y_{k}\right)}^{-\lambda_{1}}}\right]. \end{array}$$

Corresponding to *π*(*λ*_1_, *λ*_2_, *β*), the partial derivatives are

(13) $$\begin{array}{c} \frac{\partial }{\partial \lambda_{1}}\pi \left(\lambda_{1},\lambda_{2},\beta \right)=\frac{n}{\lambda_{1}}-\sum_{k=1}^{n}\log\left(1+\lambda_{2}y_{k}\right)+\sum_{k=1}^{n}\frac{\log\left(\beta \right)\log\left(\beta^{\left(1+\lambda_{2}y_{k}\right)}\right)\beta^{{\left(1+\lambda_{2}y_{k}\right)}^{-\lambda_{1}}}}{\left[\beta -\log\left(\beta \right)\beta^{{\left(1+\lambda_{2}y_{k}\right)}^{-\lambda_{1}}}\right]},\\ \frac{\partial }{\partial \beta }\pi \left(\lambda_{1},\lambda_{2},\beta \right)=\frac{n}{\lambda_{2}}-\left(\lambda_{1}+1\right)\sum_{k=1}^{n}\frac{y_{k}}{\left(1+\lambda_{2}y_{k}\right)}+\lambda_{1}\sum_{k=1}^{n}\frac{y_{k}{\left(\log\left(\beta \right)\right)}^{2}\beta^{{\left(1+\lambda_{2}y_{k}\right)}^{-\lambda_{1}}}{\left(1+\lambda_{2}y_{k}\right)}^{-\lambda_{1}-1}}{\left[\beta -\log\left(\beta \right)\beta^{{\left(1+\lambda_{2}y_{k}\right)}^{-\lambda_{1}}}\right]},\\ \frac{\partial }{\partial \lambda_{2}}\pi \left(\lambda_{1},\lambda_{2},\beta \right)=\sum_{k=1}^{n}\frac{1-\beta^{{\left(1+\lambda_{2}y_{k}\right)}^{-\lambda_{1}-1}}\left(\log\left(\beta \right){\left(1+\lambda_{2}y_{k}\right)}^{-\lambda_{1}}+1\right)}{\left[\beta -\log\left(\beta \right)\beta^{{\left(1+\lambda_{2}y_{k}\right)}^{-\lambda_{1}}}\right]}. \end{array}$$

Equating the expressions (∂/∂*λ*_1_)*π*(*λ*_1_, *λ*_2_, *β*), (∂/∂*λ*_2_)*π*(*λ*_1_, *λ*_2_, *β*), and (∂/∂*β*)*π*(*λ*_1_, *λ*_2_, *β*) to zero, i.e., (∂/∂*λ*_1_)*π*(*λ*_1_, *λ*_2_, *β*)=(∂/∂*λ*_2_)*π*(*λ*_1_, *λ*_2_, *β*)=(∂/∂*β*)*π*(*λ*_1_, *λ*_2_, *β*)=0 and solving these equations provide the estimators of *λ*_1_, *λ*_2_, and *β*, respectively.

### 4.3. An Application to YouTube Advertising Data

This subsection deals with the application of the HTBPT-Lomax model using a data set related to the YouTube advertising data. The data are available at https://www.businessofapps.com/data/youtube-statistics/. The box plot of the YouTube advertising data is provided in Figure 6 whereas the basic measures (BMs) of the data are presented in Table 3.

The HTBPT-Lomax model is compared with the Lomax model and a prominent version of the Lomax model called exponentiated Lomax (E-Lomax) model. The CDF of the E-Lomax is

(14) $$\begin{array}{c} U\left(y;\theta ,\xi \right)={\left(1-{\left(1+\lambda_{2}y\right)}^{-\lambda_{1}}\right)}^{\theta },\;5y\geq 0,\lambda_{1},\lambda_{2},\theta >0. \end{array}$$

For assessing the best fitting capability of the HTBPT-Lomax and other competitors, certain discrimination measures (DMs) and goodness-of-fits tests with respective *p* value are considered. The DMs are given by

(i) The AIC (Akaike information criterion):
  (15) $$\begin{array}{c} \text{AIC}=2k-2\Delta . \end{array}$$
(ii) The CAIC (corrected Akaike information criterion):
  (16) $$\begin{array}{c} \text{CAIC}=\frac{2kn}{n-k-1}-2\Delta . \end{array}$$
(iii) The BIC (Bayesian information criterion):
  (17) $$\begin{array}{c} \text{BIC}=k\;\log\left(n\right)-2\Delta . \end{array}$$
(iv) The HQIC (Hannan–Quinn information criterion):
  (18) $$\begin{array}{c} \text{HQIC}=2k\;\log\left(\log\left(n\right)\right)-2\Delta , \end{array}$$
where Δ represents the log-likelihood function. The other statistical tests are given by
(v) The AD (Anderson–Darling) test statistic:
  (19) $$\begin{array}{c} \text{AD}=-n-\frac{1}{n}\sum_{l=1}^{n}\left(2l-1\right)\left[\log\;P\left(y_{l}\right)+\log\left\{1-P\left(y_{n-l+1}\right)\right\}\right]. \end{array}$$
(vi) The CM (Cramér–von Mises) test statistic:
  (20) $$\begin{array}{c} \text{CM}=\frac{1}{12n}+\sum_{l=1}^{n}{\left[\frac{2l-1}{2n}-P\left(y_{l}\right)\right]}^{2}. \end{array}$$
(vii) The KS (Kolmogorov–Smirnov) test statistic:
  (21) $$\begin{array}{c} \text{KS}=\sup_{y}\left[P_{n}\left(y\right)-P\left(y\right)\right]. \end{array}$$

For certain data, a model with larger *p* value and smaller statistical tests values represents the best fit to those data.  Table 4 offers the MLEs of the models applied to the YouTube advertising data. The values of the DMs and statistical tests are listed in Tables 5 and 6, respectively. From Tables 5 and 6, we observe that the HTBPT-Lomax model is the best among the fitted models as it has the smallest values of the DMs and statistical tests and larger *p* value. This fact shows the importance of the HTBPT-Lomax distribution to deal with the data related to financial events.

In addition to the numerical results provided in Tables 5 and 6, a visual display of the competing models is provided in Figures 7 and 8. For this activity, we plotted the probability-probability (P-P) and Q-Q functions of the fitted distributions (HTBPT-Lomax (red line), Lomax (blue line), and E-Lomax (green line) (see Figures 7 and 8).

## 5. Concluding Remarks

This research studied the relationship between social media marketing and sales. In this paper, we studied the effect of YouTube advertising on the sales and profit. The data and information were scientifically tested and analyzed. For scientific study and analysis, we considered a linear regression modeling approach along with two statistical tests such as *t*-test and *F*-test. Based on these tools, it is observed that there was a positive relationship between YouTube advertising and sales. Besides these tests, the correlation test was also performed, and it found that there is a positive correlation between YouTube advertising and sales. A positive correlation means that the more we spend money on the YouTube advertising, the more will be sales and profit. Finally, the HTBPT-Lomax distribution was applied to model the YouTube advertising data. Based on the certain statistical tools, it is showed that the HTBPT-Lomax model outclassed the competitors.

## Figures and Tables

**Figure 1:** Relationship between YouTube advertising and sales.

**Figure 2:** Graphical representations of the residuals.

**Figure 3:** Box plot and Cook's distance plot of the YouTube advertising data.

**Figure 4:** Graphical representations of the residuals.

**Figure 5:** Different plots of *p*(*y*; *β*, *ξ*).

**Figure 6:** The box plot of the YouTube advertising data.

**Figure 7:** The P-P plots of the HTBPT-Lomax, Lomax, and E-Lomax models.

**Figure 8:** The Q-Q plots of the HTBPT-Lomax, Lomax. and E-Lomax models.

**Table 1:** Numerical results of SLRM based on *t*-test.

Adv. media	RCs	Estimated values	SE	*t*-statistic	Pr(>|*t*|)
YouTube	*β*_0_	4.84707	0.39901	12.14700	2*e* − 16
	*β*_1_	0.04801	0.00482	9.95900	2*e* − 16

**Table 2:** Numerical results of SLRM based on *F*-test.

Adv. media	*R* ^2^	Adjusted *R*^2^	*F*-statistic	*p* value	Degree of freedom
YouTube	0.4366	0.4322	99.18	2.2*e* − 16	1 and 128

**Table 3:** The BMs of the YouTube advertising data.

Minimum	1st quartile	Median	Mean	3rd quartile	Maximum
8.79	88.09	156.00	160.26	243.21	352.75

**Table 4:** The estimated values of the parameters corresponding to the YouTube advertising data.

Model	*λ*_1_	*λ*_2_	*β*	*θ*
HTBPT-Lomax	40.19293	0.01498	0.02453	—
Lomax	37.76721	0.00834	—	—
E-Lomax	40.94021	0.01188	—	2.11716

**Table 5:** The DMs of the fitted models corresponding to the YouTube advertising data.

Model	AIC	CAIC	BIC	HQIC
HTBPT-Lomax	530.80220	530.99260	539.40480	534.29770
Lomax	569.18910	569.28360	574.92420	571.51950
E-Lomax	540.77130	540.96180	549.37390	544.26680

**Table 6:** The analytical measures of the fitted models corresponding to the YouTube advertising data,.

Model	AD	CM	KS	*p*-value
HTBPT-Lomax	0.30471	2.12335	0.09510	0.19030
Lomax	0.42388	2.83853	0.19251	0.13070
E-Lomax	0.46870	3.10789	0.10482	0.11490

## Data Availability

The data set is available from the corresponding author upon request.

## Appendix

The *R* − Code used for analysis under Section 5 is as follows:

*y* {\textless}-read.csv (file.choose (), header = TRUE)
*y* = *y* [, 1]
*y* = *y* [!is.na (*y*)]
  data = *y*
  data
  %-----------------------------------------------------------------
  %-------------- PDF
  %-----------------------------------------------------------------
  pdf_Rayleigh {\textless}-function (par, *x*)
  {
  Lambda1 = par [1]
  Lambda2 = par [2]
  beta = par [3]
  Lambda1*∗*Lambda2*∗*((1 + Lambda2*∗y*)^(-Lambda1-1))*∗*
  (beta-(log (beta))*∗*(beta^((1 + Lambda2*∗*y)^(-Lambda1))))
  }
  %-----------------------------------------------------------------
  %-------------- CDF
  %-----------------------------------------------------------------
  cdf_pm {\textless}- function (par, x)
  {
  Lambda1 = par [1]
  Lambda2 = par [2]
  beta = par [3]
  (beta^((1 + Lambda2*∗y*)^(-Lambda1)))-beta*∗*((1 + Lambda2*∗y*)^(-Lambda1))
  }
  set.seed (0)
  goodness.fit (pdf = pdf_pm, cdf = cdf_pm,
  starts = *c* (0.5, 0.5, 0.5), data = data,
  method = “BFGS,” domain = *c* (0, Inf), mle = NULL)
